# Hepcidin: regulation of the master iron regulator

**DOI:** 10.1042/BSR20150014

**Published:** 2015-05-19

**Authors:** Gautam Rishi, Daniel F. Wallace, V. Nathan Subramaniam

**Affiliations:** *The Membrane Transport Laboratory, The QIMR Berghofer Medical Research Institute and School of Medicine, University of Queensland, Brisbane, Queensland 4006, Australia

**Keywords:** erythropoiesis, hepcidin, hypoxia, inflammation, iron, ACD, anaemia of chronic disease, ATOH8, atonal homologue 8, BMP, bone morphogenetic protein, BMPR, BMP receptor, CREB/H, cAMP response element-binding protein/H, EGF, epidermal growth factor, EPO, erythropoietin, ERFE, erythroferrone, FPN, ferroportin, GDF15, growth differentiation factor 15, HEK, human embryonic kidney, HFE, haemochromatosis protein, HGF, hepatocyte growth factor, HH, hereditary haemochromatosis, HIF, hypoxia-inducible factor, HJV, haemojuvelin, HRE, hypoxia-responsive element, HSC, hepatic stellate cell, IL, interleukin, IRIDA, iron refractory iron deficiency anaemia, JAK, Janus kinase, KC, Kupffer cell, LPS, lipopolysaccharide, LSEC, liver sinusoidal endothelial cell, mTOR, mammalian target of rapamycin, NPC, non-parenchymal cell, PDGF-BB, platelet-derived growth factor-BB, PHD, prolyl dehydrogenase, pSMAD1/5/8, phospho-SMAD1/5/8, sHJV, soluble HJV, SMAD, sma and mothers against decapentaplegic homologue, STAT, signal transducer and activator of transcription, TF, transferrin, TFR, transferrin receptor, TGF-β, transforming growth factor-β, Tmprss, transmembrane protease, serine, TNF, tumour necrosis factor, TWSG1, twisted gastrulation BMP signalling modulator 1, VHL, von Hippel-Lindau

## Abstract

Iron, an essential nutrient, is required for many diverse biological processes. The absence of a defined pathway to excrete excess iron makes it essential for the body to regulate the amount of iron absorbed; a deficiency could lead to iron deficiency and an excess to iron overload and associated disorders such as anaemia and haemochromatosis respectively. This regulation is mediated by the iron-regulatory hormone hepcidin. Hepcidin binds to the only known iron export protein, ferroportin (FPN), inducing its internalization and degradation, thus limiting the amount of iron released into the blood. The major factors that are implicated in hepcidin regulation include iron stores, hypoxia, inflammation and erythropoiesis. The present review summarizes our present knowledge about the molecular mechanisms and signalling pathways contributing to hepcidin regulation by these factors.

## Abstract 2

Hepcidin, the central regulator of iron homoeostasis, is itself regulated by many factors including iron stores, hypoxia, inflammation and erythropoiesis. The present review summarizes our present knowledge about the molecular mechanisms and signalling pathways contributing to hepcidin regulation.

## HEPCIDIN

Iron is an essential element for many biological processes and hence it is required for the survival of all living organisms. Iron can also be toxic in excess and its misregulation is the basis for many clinical disorders. Soon after its identification in 2000, it was realized that the liver-expressed peptide hepcidin plays a central role in the systemic regulation of iron metabolism; its imbalance or aberrant expression was found to be at the centre of many iron disorders. Aptly, it has been described as the master regulator of iron metabolism and the iron regulatory hormone.

Hepcidin was originally identified as a liver-expressed antimicrobial peptide (LEAP1) with direct antimicrobial activity against a number of bacterial and fungal species [1,2]. It was soon discovered that hepcidin plays a major role in the regulation of iron homoeostasis, being overexpressed in the livers of mice with an induced (dietary or parenteral) iron overload [3]. Disruption of the gene in mice also resulted in iron overload, further confirming its importance in iron metabolism [4]. Hepcidin acts as a negative regulator of iron stores; in response to increased iron levels, the liver increases hepcidin synthesis which then acts on the sites of absorption (enterocytes of the duodenum), storage (primarily hepatocytes of the liver) or recycling (macrophages of the reticuloendothelial system) leading to a decrease in the release of iron from these tissues.

Hepcidin exerts its influence by binding to and inducing the internalization and degradation of ferroportin (FPN), the only known exporter of iron [5]. Given that iron plays an important role in a variety of cellular, metabolic and physiological processes, it is not surprising that hepcidin itself is regulated in response to a wide range of external and internal stimuli. Some of the best studied of these stimuli include tissue iron stores, transferrin (TF) saturation, hypoxia and inflammation. In addition, it is also known that the erythropoietic demand reduces hepcidin levels to increase iron availability for the production of red blood cells, but the molecular details of this mechanism are still to be deciphered [6].

## IRON REGULATORY DISORDERS AND HEPCIDIN

Either too little or too much iron can have detrimental effects on health, leading to iron deficiency anaemia on the one hand and iron overload or haemochromatosis on the other. Hereditary haemochromatosis (HH) is caused by mutations in genes involved in the regulation of iron metabolism, resulting in excess iron accumulation in tissues and consequent damage, manifesting as fatigue, liver disease, diabetes mellitus, arthropathy, hypogonadism and/or cardiomyopathy [7]. The gene encoding HFE (haemochromatosis protein) is mutated in the majority of patients with HH (type 1 [8]). Two juvenile forms of HH have been described that are caused by mutations in the genes encoding haemojuvelin (HJV) (*HFE2*; type 2A) [9] or hepcidin itself (*HAMP*, hepcidin anti-microbial peptide; type 2B) [10]. Another adult onset form of HH (type 3) is caused by mutations in the gene encoding TF receptor 2 (*TFR2*) [11]. An autosomal dominant form of iron overload is caused by mutations in the gene encoding the iron exporter and hepcidin receptor FPN (*SLC40A1*, solute carrier family 40 member 1) [12,13]. All these forms of iron overload can be attributed to defects or imbalances in the hepcidin–FPN axis that controls iron homoeostasis leading to iron overload. Anaemia can also be caused by imbalances in the hepcidin–FPN axis. For example, a form of iron refractory iron deficiency anaemia (IRIDA) can be caused by mutations in the gene encoding matriptase-2 [transmembrane protease, serine 6 (*TMPRSS6*)], a negative regulator of hepcidin [14–16]. The anaemia of chronic disease (ACD) has also been linked to increased expression of hepcidin [17]. The study of these iron-associated disorders has greatly increased our understanding of how iron homoeostasis and hepcidin are regulated and the signalling pathways involved.

In the following sections, we review the known and potential signalling pathways and molecules that influence hepcidin synthesis and hence iron metabolism.

## POSITIVE REGULATORS OF HEPCIDIN

The two major stimuli that are known to increase hepcidin synthesis in the liver are body iron status and inflammation.

### Iron-mediated hepcidin regulation

#### The BMP–SMAD pathway

The high expression of hepcidin in hepatocytes and studies into its regulation has pin-pointed the liver as the control centre for the regulation of systemic iron homoeostasis. The most commonly studied pathway that influences hepcidin transcription in response to an increase in body iron levels is the bone morphogenetic protein (BMP)–sma and mother against decapentaplegic (SMAD) pathway. BMPs belong to the transforming growth factor-β (TGF-β) superfamily of cytokines. They have been shown to play crucial roles in development, cell proliferation, cell differentiation and apoptosis. It is now well established that the BMP–SMAD pathway has a central role in the regulation of hepcidin in response to body iron levels [18].

The link between the SMAD pathway and iron metabolism was discovered when it was shown that mice with hepatocyte-specific deletion of *Smad4*, develop severe iron overload [19]. The livers of these mice had a 100-fold suppression of *Hamp* mRNA levels, suggesting that SMAD4 is involved in the transcriptional regulation of *Hamp* [19]. It was proposed that the TGF-β–BMP pathway was involved in hepcidin regulation, as wild-type hepatocytes showed an increase in *Hamp* mRNA levels in response to treatment with TGF-β or BMP4, whereas this response was abrogated in *Smad4^−/−^* hepatocytes [19].

More recently it has been shown in mice that BMP6 is the predominant BMP ligand responsible for hepcidin regulation *in vivo* [20–22]. Initially it was shown that in mice the *Bmp6* transcript was regulated similarly to hepatic *Hamp* in response to different dietary iron conditions [20]. Subsequent studies demonstrated that *Bmp6* null mice develop a rapid and massive accumulation of iron in the liver that is related to a marked reduction in liver *Hamp* expression [21,22]. It was also shown that the nuclei of the hepatocytes of *Bmp6* null mice had less phospho-SMAD1/5/8 (pSMAD1/5/8) compared with wild-type mice fed a control diet or an iron-enriched diet [21], indicating that it is a defect in the BMP–SMAD signalling pathway that is responsible for reduced hepcidin transcription. Mice treated with BMP6 showed a dose-dependent reduction in serum iron and TF saturation along with an increase in hepatic *Hamp* expression, further supporting the concept that BMP6 is required for proper *Hamp* regulation [22].

#### Molecules involved in BMP–SMAD-mediated regulation of hepcidin

A major breakthrough was made when it was shown that HJV, the protein mutated in the majority of cases of juvenile HH, acts as a BMP co-receptor [23]. This confirmed the role of HJV in hepcidin regulation and was consistent with reports showing that patients with type 2A HH had low hepcidin levels [9]. It was also shown that HJV acted through the BMP pathway rather than the TGF-β pathway since the presence or absence of HJV did not affect the activity of a TGF-β responsive promoter element [23]. Hepatocytes lacking HJV had a blunted response to BMP2 treatment, indicating that HJV acts through or plays a role in the BMP–SMAD signalling pathway [23]. Using primary hepatocytes from mice and a hepatoma cell line, it was shown that BMP2, 4 and 9 can induce hepcidin transcription independently of *Hfe*, *Tfr2* or *Il6* (interleukin 6). It was also suggested that BMP9 is the most potent stimulator of hepcidin [24]. Treatment of mice with BMP2 also lowered hepcidin expression in the liver and serum iron levels [25]. These results suggested that BMP–SMAD signalling is an important pathway in the regulation of iron homoeostasis.

The suggestion that the liver-expressed Tmprss6 acts as an upstream regulator of the BMP–SMAD pathway added another layer to this complex regulatory pathway [26]. Patients and mice with mutations in the *TMPRSS6* gene develop IRIDA. It was demonstrated that the cause of this anaemia is high levels of hepcidin [14–16]. Silvestri et al. [26] showed that matriptase-2 cleaved HJV and consequently suppressed signalling through the BMP–SMAD pathway resulting in reduced transcription of *Hamp*. In a recent study, it was shown that decreased intracellular iron levels lead to an increase in TMPRSS6 protein levels in HepG2 cells [27]. TMPRSS6 protein levels increased due to a decrease in the lysosomal-mediated degradation of the protein and not due to increased *Tmprss6* mRNA levels [27]. These results suggest a novel iron-mediated regulation of TMPRSS6 protein.

The liver is thought to be the centre for systemic iron regulation and it is believed to mediate this regulation by modulating the amount of *HAMP* produced in response to body iron status. The control of hepcidin expression involves molecules that can sense the circulating levels of iron and relay these messages through signal transduction pathways to the nucleus to regulate hepcidin transcription. Thought to be central to this iron sensing mechanism are the HH-related proteins HFE and TFR2 and the classical TFR1. It has been suggested that the interactions between these molecules are important for cells to sense the levels of holo-TF. Early studies linked HFE, an atypical MHC (major histocompatibility complex) class I protein to iron metabolism by identifying an interaction with TFR1 [28,29]; however, the mechanism responsible for regulating iron homoeostasis was not immediately apparent. With increasing levels of holo-TF, HFE is displaced from the HFE–TFR1 complex, a step thought to be important for initiating a signalling cascade that results hepcidin transcription [30].

The interaction of HFE with TFR1 has been well characterized and the domains and amino acids responsible for this interaction have been mapped [28,31]. Initial studies failed to detect an interaction between the extracellular domains of human HFE and TFR2 [32]. However, later work, involving overexpression of HFE and TFR2 in cell lines was able to detect an interaction between these two proteins [33,34]. The formation of a multi-protein complex (consisting of HFE, TFR2, HJV) at the surface of the hepatocytes has also been suggested [35]. In contrast with these studies, other studies using *Hfe^−/−^*–*Tfr2^−/−^* double knockout mice [36] and transgenic mice overexpressing myc-tagged *Hfe* [37] have suggested that HFE and TFR2 need not interact to regulate hepcidin synthesis. In support of this, using the recently developed proximity ligation assay, we also failed to detect an interaction between these two proteins, in a mouse hepatoma cell line stably expressing both HFE and TFR2 [38].

HFE and TFR2 are also thought to modulate hepcidin expression through pathways related to BMP–SMAD. *Hfe^−/−^* mice and humans with *HFE*-related HH have been shown to have deficiencies in BMP–SMAD signalling despite appropriately increased levels of BMP6 [39–41]. These studies suggested that HFE is involved in modulating BMP–SMAD signalling downstream of BMP6. Consistent with this, a recent study demonstrated that HFE interacts with the BMP type I receptor ALK3 (activin-like kinase 3), stabilizing the protein at the cell surface and enhancing BMP signalling to increase hepcidin expression [42]. TFR2 deficient mice have also been shown to have reduced levels of pSMAD1/5/8 in the liver suggesting that TFR2 also modulates the BMP–SMAD pathway to regulate hepcidin [43]. It was recently suggested that TFR2 is involved in the up-regulation of BMP6 by iron and that inappropriately low BMP6 levels in *Tfr2^−/−^* mice may be responsible for reduced BMP–SMAD signalling and low hepcidin [44]. On the basis of these recent advances, we propose a new model for the roles of HFE and TFR2 in the regulation of *HAMP*. In response to increased TF saturation TFR2 initiates a signalling cascade which results in the synthesis of *BMP6*. BMP6 protein is then secreted and interacts with the BMP receptors (BMPRs). HFE is required to transport BMPR type I to the surface and hence is required for the proper interaction between BMPs and their receptors. In the absence of a functional TFR2, BMP6 is not produced appropriately in response to increased iron levels and hence results in an inappropriate *HAMP* response. In the absence of a functional HFE, the type I BMPR is not properly localized to the surface of hepatocytes resulting in impaired SMAD signalling and hence inappropriately low *HAMP* levels.

There appear to be more than one pathway involved in regulation of hepcidin in response to iron levels [45]. The response to acute and sudden changes in TF saturation (extracellular iron) seems to involve HFE and TFR2 which presumably sense the levels of TF saturation and increase the sensitivity of BMPRs to iron levels [45]. In response to chronic dietary iron overload *Hfe^−/−^*, *Tfr2^−/−^*, *Bmp6^−/−^* and *Hjv^−/−^*, mice showed an increase in hepcidin mRNA levels [45]. This suggests that in addition to BMP signalling there could be other pathways involved in regulating hepcidin levels in response to intracellular iron levels [45].

#### Regulation of BMP6

In recent years, the BMP–SMAD pathway has been demonstrated as the predominant pathway responsible for regulating *HAMP* in response to iron. Although there have been a number of studies defining the role of this pathway in the regulation of iron metabolism, the molecular details of how an increase in iron levels induce *Bmp6* are not known. The liver is a heterogeneous organ composed of different cell types of which hepatocytes form approximately 70% of the cells and the rest comprise non-parenchymal cells (NPCs), including liver sinusoidal endothelial cells (LSECs), hepatic stellate cells (HSCs), Kupffer cells (KCs) and other cells [46]. It has been suggested that in hepatocytes BMP6 levels correlate with iron stores [47] and are not regulated by serum iron or TF saturation.

A growing body of evidence suggests a more complicated regulation of BMP6 in response to increases in iron. It was recently suggested that BMP6 expression in response to serum iron is mediated by the NPCs [48] and that ferritin may also be involved [49]. *Bmp6* transcript was predominantly produced in the NPCs, especially the LSECs and HSCs, indicating that BMP6 could be acting in a paracrine fashion to influence *Hamp* transcription in neighbouring hepatocytes [48].

A few studies have showed that primary hepatocytes can respond to holo-TF treatment [50,51] whereas in previous experiments primary hepatocytes and immortalized hepatocyte cell lines did not up-regulate hepcidin in response to holo-TF treatment [17,52]. Results from these and others studies [53,54] have pointed to an interaction between different cell types in the liver. Sasaki et al. [26] previously showed that when the human hepatoma-derived cell line HepG2 was co-cultured with the human macrophage cell line THP1 (Tamm-Horsfall protein 1) (with or without contact), they could induce production of HAMP in response to holo-TF treatment.

These studies suggest that the ‘iron sensing’ role of the liver could in fact be a function of multiple cell types: the NPCs and the hepatocytes may sense the iron levels and respond by releasing BMP6, which then initiates a cascade of events in hepatocytes leading to the production of hepcidin. This intercellular cross-talk seems to be one of the mechanisms mediating *Bmp6* up-regulation in response to iron, but the actual molecular pathways underlying the production of BMP6 in response to either serum iron or liver iron stores still remain to be identified.

### Inflammatory regulation of hepcidin

The second major signalling pathway known to play a role in the regulation of *HAMP* transcription is the JAK (Janus kinase)–STAT3 (signal transducer and activator of transcription 3) pathway; the stimulus for this regulation coming mainly through inflammatory cytokines.

#### Inflammation and iron metabolism

It was known that serum iron levels can be lower in patients with chronic inflammation and that this can lead to the ACD. The first insight into how this could be mediated was provided by the discovery of hepcidin's role in iron metabolism, where Pigeon et al. [3] showed that treatment of hepatocytes with lipopolysaccharide (LPS) led to an increase in *Hamp* levels [3]. Subsequently, using human primary hepatocytes, it was shown that HAMP is a type II acute phase protein, as it was induced by treatment with interleukin 6 (IL6) but not with cytokines involved in the type I response including tumour necrosis factor-α (TNF-α) or IL1α [17,55]. Further studies established that this response to inflammatory signals is not mediated by the KCs in the liver, where even after depletion of KCs the liver was able to increase hepcidin in response to IL6 treatment [56]. Evidence that the *HAMP* promoter contains a STAT3-binding site provided further evidence for the mechanism of *HAMP* regulation during inflammation [57]. Pietrangelo et al. [58], using transgenic mice in which the main IL6–gp130 (glycoprotein 130 kD) signalling pathways have been disrupted, confirmed that STAT3 was the primary transcription factor that mediates the IL6 induction of hepcidin [58]. The JAK–STAT3 pathway works in a similar way to the BMP–SMAD pathway, where the binding of a cytokine ligand, for example IL6, to the receptor induces a signalling cascade which results in the phosphorylation of STAT3 [59]. The phosphorylated STAT3 is then translocated to the nucleus where it binds to tissue-specific transcription factors and cofactors to mediate the transcriptional activation or repression of target genes [59]. Previously, using a transgenic mouse model with hepatocyte-specific deletion of STAT3 it was shown that the hypoferremic response to inflammation, involving hepcidin induction, is mediated directly through hepatocytes rather than involving other cell types [60].

The increase in hepcidin levels in response to infection seems to have evolved as a defence mechanism to protect the host from infections. Most micro-organisms require iron for their growth and proliferation, hence limiting the release of iron into the blood by increasing the levels of hepcidin would result in restricted iron availability to the infectious agent. Indeed some previous studies have shown results which support this hypothesis. It has been shown by our laboratory that increased iron stores result in a worse disease outcome in schistosomiasis [61] and that iron deficiency leads to better survival rates in children with malaria [62]. It was shown that in children, iron deficiency decreased the prevalence of parasitaemia and severe malaria. These results have initiated a new discussion about the treatment of patients suffering from the ACD, although the negative consequences of anaemia can be detrimental to the health of the patients, iron therapies to counteract iron deficiency may support the pathogen and lead to worse pathology, hence warranting a closer and more careful monitoring of such patients.

It has been suggested that there is some interaction/cross-talk between the BMP–SMAD and the JAK–STAT pathway. Mice lacking SMAD4 in the hepatocytes did not show an increase in hepcidin mRNA levels when treated with IL6, suggesting that the inflammation- and iron-mediated pathways of hepcidin regulation may intersect at SMAD4 [19]. Subsequently, it was shown that human hepatoma cell lines, zebrafish and mice pre-treated with a BMP type I receptor inhibitor had a reduced hepcidin response to IL6 treatment [63]. Recently, it was shown that the BMP type I receptor Alk3 is required for an IL6-mediated hepcidin response [64]. Mice lacking Alk 3 were unable to increase hepcidin mRNA levels or reduce serum TF saturation in response to an overexpression of IL6 (injection of adenovirus expressing IL6) or injection of recombinant murine IL6 [65].

LPS treatment of mice increased SMAD phosphorylation similarly in the wild-type and *Bmp6^−/−^* mice [66]. This up-regulation of pSMAD1/5/8 levels does not seem to work through any of the BMP ligands as the mRNA levels of *Bmp2, Bmp4, Bmp5, Bmp6, Bmp7* and *Bmp9* did not differ between the control and LPS challenged mice [66]. The mRNA levels of another TGF-β superfamily member activin B were shown to be increased in the animals treated with LPS [66]. Treatment of human hepatoma cells and mouse primary hepatocytes with activin B induced an increase in hepcidin mRNA and pSMAD1/5/8 levels [66]. These observations suggest that activin B could be the BMP ligand involved in the cross-talk between the BMP–SMAD pathway and inflammation-mediated regulation of hepcidin [66].

There is some evidence suggesting cross-talk between the iron sensing and the inflammatory pathways regulating hepcidin. Initially it was shown that HFE is required to mediate the inflammatory hepcidin response, as HFE-deficient mice were unable to increase hepcidin in response to LPS [67]. Later studies contradicted this and suggested that HFE is not required for the LPS- and IL6-mediated increase in hepcidin transcription [68,69]. In a previous study published by our laboratory, it was shown that mice lacking *Tfr2* or both *Tfr2* and *Hfe* have a decreased hypoferremic response after LPS injection [70]. Although these mice could elevate hepcidin in response to LPS, the inadequate hypoferremic response was attributed to lower levels of basal hepcidin.

## NEGATIVE REGULATORS OF HEPCIDIN

Physiological processes like erythropoiesis, which require a constant supply of iron, act as negative regulators of hepcidin. Repression of *HAMP* is a mechanism to make more iron available in order to maintain normal homoeostasis.

### The erythroid control of hepcidin

One of the most important functions of iron is as an essential component of the oxygen transporting proteins haemoglobin and myoglobin. Iron is crucial for the formation and maturation of red blood cells (erythropoiesis). Anaemia caused by dietary iron deficiency is one of the most common nutritional disorders in the world. This requirement for iron suggests that erythropoiesis itself could be involved in regulating the amounts of bioavailable iron in the circulation. This was shown to be the case in mouse studies, where, the suppression of erythropoiesis by irradiation or post-transfusion polycythaemia dramatically increased the levels of hepcidin, indicating that erythropoiesis could suppress *Hamp* expression [71]. Physiologically, this would be important for the body in cases of haemorrhage or haemolysis, where there is a rapid loss of blood and subsequently a huge increase in the demand for iron to produce more red blood cells to alleviate the condition. In such a situation an increased influx of iron from the gut and release of iron from the macrophages and liver stores would be required to keep up with erythropoietic demand. This can only be maintained if the physiological levels of *Hamp* are kept low. This erythroid regulation of *Hamp* synthesis is believed to override the regulation by iron stores, as seen in patients with iron loading anaemias like thalassaemia, where dysregulated erythropoeisis is able to suppress *Hamp* even in the presence of iron overload. This suggests that the proposed ‘erythroid regulator’ [72], which supposedly maintains iron levels in response to erythropoietic demand exerts its influence by modulating the levels of hepcidin.

#### Erythropoietin and hepcidin

One of the main signalling molecules which mediate erythropoiesis is erythopoietin (EPO); it is produced mainly in the kidney and is required for proper erythropoiesis, as it helps in the maturation and development of erythroblasts in the later developmental stages. When human subjects were treated with EPO the levels of circulating hepcidin decreased abruptly within 24 h with the maximal suppression at 72 h, this showed that EPO can influence hepcidin [73]. In mice treated with inhibitors of erythropoiesis, increases in EPO levels or treatment with PHZ (phenylhydrazine) does not lead to a suppression of *Hamp* [74,75]. These results suggested that although EPO can regulate *HAMP*, it does not act directly and therefore cannot be the long sought after erythroid regulator.

#### The erythroid regulator

It was hypothesized that this erythroid factor is a molecule secreted by erythroblasts [76]. Microarray analyses of primary human erythroblasts were performed to identify the molecules that respond to this increased demand [76]. These studies identified two potential erythroid regulators, growth differentiation factor 15 (GDF15) [76] and twisted gastrulation BMP signalling modulator 1 (TWSG1) [77]. GDF15 levels in patients suffering from symptomatic β-thalassaemia were significantly higher than normal controls [76]. On treating primary human hepatocytes or HuH7 cells with high concentrations of GDF15 (similar to those found in patients with thalassaemia) hepcidin transcription was inhibited [76]. Similarly hepcidin was repressed in cells cultured in sera from thalassaemic patients [76]. TWSG1 was also shown to inhibit hepcidin synthesis in HuH7 cells and primary human hepatocytes by inhibiting BMP–SMAD signalling [77]. Based on these two studies and the expression pattern of the two molecules a model was proposed for the inappropriate erythroid regulation of hepcidin in thalassaemia, where TWSG1 (produced in the early erythroblasts) acts indirectly by inhibiting the BMP–SMAD pathway and GDF15 which is produced in late erythroblasts acts directly to inhibit hepcidin, although the signalling mechanism is unknown [77].

Subsequently it was shown that *Gdf15* knockout mice subjected to two consecutive phlebotomies did not show any differences in hepcidin levels as compared with the wild-type mice, these results suggested that either GDF15 is not the putative erythroid factor or its effects can be overcome by other pathways involved in hepcidin regulation [78].

The most recent addition to the list of potential erythroid regulators is the product of the *Fam132b* gene, referred to as erythroferrone (ERFE) [79]. This molecule is also known as myonectin or C1q/TNF-related protein family member 15 (CTRP15) [79]. ERFE has been proposed to be a stress-erythropoeisis specific erythroid regulator of hepcidin. Similar to GDF15 and TWSG1, ERFE is expressed in erythroblasts and after EPO treatment, the mRNA levels of *Fam132b* increase only in the erythropoietic organs of adult mice (bone marrow and spleen) [79]. Mice lacking *Fam132b* have a blunted suppression of hepcidin in response to phlebotomy as compared with wild-type mice suggesting that *Fam132b* is required for hepcidin suppression after blood loss [79]. The levels of *Fam132b* were found to be increased in mouse models of β-thalassaemia intermedia, again indicating that it could be playing a role in the suppression of hepcidin in iron loading anaemias [79]. Recent results from our laboratory using the *Tmprss6–Hfe–Tfr2* triple knockout and *Tmprss6–Tfr2* double knockout mice have shown that although *Fam132b* levels are higher in these mice, they are unable to suppress *Hamp* levels [80]. These results suggest that ERFE could be a potential erythroid regulator of *HAMP* in some conditions (thalassaemias) and not in others (IRIDA). Although these results are promising they need to be verified in human studies. The molecular mechanisms underlying the action of ERFE are still not known, although it appears that its regulation of *HAMP* is not related to the iron sensing or BMP–SMAD signalling pathway [79].

### Hypoxia and hepcidin axis

The main function of the iron in haemoglobin is to bind oxygen; hence the levels of tissue oxygen depend on the availability of iron to form haemoglobin. It has long been known that hypoxic conditions increase erythropoeisis and hence enhance oxygen availability. Similar to erythropoeisis it was shown that *HAMP* levels decrease in hypoxic conditions [81].

#### Hypoxia-inducible factors and hepcidin regulation

The main mediator of the hypoxic regulation of genes is the transcription factor hypoxia-inducible factor (HIF). There are three known subunits of HIF: HIF1α, HIF2α and HIF3α. In the presence of oxygen, these subunits are modified by prolyl dehydrogenase (PHD) and subjected to proteasomal degradation by a tumour suppressor, von Hippel-Lindau (VHL) factor [82]. In oxygen-deprived conditions, PHD is inactivated leading to stabilization of the HIF subunits [82]. The subunits then translocate to the nucleus and bind the aryl hydrocarbon nuclear receptor translocator or HIF1β (ARNT/HIF1β) forming a heterodimer. The heterodimers then binds to hypoxia-responsive elements (HREs) in the DNA and regulate hypoxia-specific target genes, one of which is *EPO.*

The first direct evidence for the involvement of HIFs in the regulation of *Hamp* was provided in mice with a hepatocyte-specific deletion of *Hif1α* [83]. Unlike wild-type mice, these mice did not show a decrease in *Hamp* in response to iron deficiency or hypoxia [83]. The levels of HIF1α in wild-type mice with iron deficiency were also shown to increase, indicating the importance of HIF1α in hypoxia-mediated repression of *Hamp* [83]. Using ChIP, it was shown that HIF1α binds to three putative HREs in the *Hamp* promoter and reduces *Hamp* expression in both human cells [human embryonic kidney (HEK)293 cells] and mouse liver tissues [83]. Using intestinal epithelial cell-specific knockouts of *Hif1α* and *Hif2α* it was demonstrated that *Hif2α* is required for iron absorption, as mice lacking *Hif2α* in the intestinal epithelium developed a marked iron deficiency, characterized by low liver and serum iron levels [84]. Interestingly, these mice also had lower liver *Hamp* as compared with the wild-type animals [84]. In contrast with these studies which showed a direct effect of the HIFα subunits on iron metabolism related proteins, another study suggested that this response is not direct [85]. Although Volke et al. [85] did get a reduction in *Hamp* levels in response to hypoxia, a knockdown of either *HIF1α, HIF2α* or both did not lead to an increase in *HAMP* levels. Interestingly, induction of hypoxia led to a decrease in *TFR2* mRNA levels and this correlated with the decrease in *HAMP* [85].

Hypoxia also increases *furin* mRNA levels through HIF1α in HepG2 and Hepa-1 (mouse hepatoma) cells [86]. Furin is a protease that was shown to cleave HJV in the endoplasmic reticulum to release soluble HJV (sHJV) [87]. sHJV is thought to be an antagonist to the BMP–SMAD regulation of hepcidin; it acts by binding to the BMPs and reducing the receptor–ligand interaction both *in vivo* and *in vitro* [25]. Silvestri et al. [87] also showed that the levels of furin increase in hypoxic and iron-deficient conditions and hypothesized that this could be one of the indirect mechanisms of hypoxia-mediated *Hamp* repression. Hypoxia was also shown to regulate the levels of *TMPRSS6*, which as discussed above, is a negative regulator of BMP–SMAD signalling [88]. In hypoxic or iron-deficient conditions, the levels of *TMPRSS6* mRNA increased in Hep3B cells, but this increase was not observed in cells where *HIF1α* was knocked down, suggesting that this could be another indirect effect of HIF1α [88].

Using a hepatocyte-specific *Hif2α* knockout mouse, it was shown that in conditions of iron-deficiency HIF2α is not required for the repression of hepcidin, however mice with a constitutively active HIF2α (*Vhlh/Hif1α* double knockout mice) had lower hepcidin levels in their livers [89]. Contrary to the results shown by Silvestri et al. [87] and Lakhal et al. [88], there was no change in the mRNA levels of *Tmprss6* and a decrease in the levels of *furin* in these mice. These results suggest that the reduction in *Hamp* mRNA levels is not due to a suppression of BMP–SMAD signalling in these mice. The authors also suggested that this repression is mediated through the increase in erythropoietic drive in the mice, as an injection of neutralizing erythropoietin serum over five consecutive days increased *Hamp* levels [89].

#### Hypoxia and growth factors

In human volunteers who were subjected to hypoxic conditions for 6 h, hepcidin levels decreased. The levels of other cytokines were also measured and surprisingly IL6 levels increased in these subjects. In addition to this, an increase in platelet-derived growth factor (PDGF)-BB was also observed [90]. There was a significant correlation between the increase in PDGF-BB and *HAMP* levels suggesting that PDGF-BB could be the hypoxic mediator of *HAMP* repression [90]. Treatment with EPO did not increase levels of PDGF-BB and treatment of normoxic and hypoxic mice with a PDGF receptor kinase inhibitor increased *Hamp* levels in mice, suggesting that hypoxia mediates this effect through the PDGF pathway [90]. The hypoxic mice did not show any changes in the levels of pSMAD1/5/8 or pSTAT3, suggesting that the increase in *Hamp* is not mediated through the BMP–SMAD or the JAK–STAT pathway [90]. Hypoxic mice exhibited a decrease in the levels of CAAT enhancer-binding protein α (C/EBPα), cyclic AMP response element-binding protein (CREB) and CREB-H [90]. Injection of PDGF-BB did not exhibit a decrease in liver hepcidin mRNA levels in the CREB-H knockout mice indicating that CREB-H is required for PDGF-BB-mediated down-regulation of hepcidin [90]. Previously CREB-H has also been suggested to play a role in endoplasmic reticulum stress-mediated induction of hepcidin [91].

These studies have added to our understanding about the effect of hypoxia on iron metabolism. It is now a widely accepted fact that hypoxia increases iron availability by reducing the levels of hepcidin. The studies mentioned above suggest that there are many potential mediators and pathways that can mediate the hypoxic repression of hepcidin. We are still unclear about the exact molecular mechanisms underlying this repression, whether it is a direct effect of hypoxia or an indirect consequence through the increased erythropoietic drive or both is still unclear. It is also unclear whether it is an effect mediated through HIF1α, HIF2α or both molecules. The observations that hypoxia can lead to a change in the transcript and protein levels of iron sensing molecules (*Tfr2*, HJV and *Tmprss6*) also points to a deeper link between hypoxia and iron metabolism.

It was also proposed that the repression of *HAMP* in conditions of hypoxia, anaemia and erythropoeisis is through a common transcription factor atonal homologue 8 (ATOH8) [92]. *ATOH8* expression in HEK293T cells increased SMAD1/5/8 phosphorylation and *HAMP* levels. Mice treated with EPO, PHZ or exposed to hypoxia for 24 or 72 h showed a decrease in *Atoh8* mRNA and protein levels [92]. Using ChIP, it was shown that ATOH8 binds to the E-box elements in the *HAMP* promoter, hence *ATOH8* can potentially regulate *HAMP* both directly (binding to the promoter) and indirectly (increasing the phosphorylation of SMAD 1/5/8 [92].

### Other mediators of *HAMP* regulation

Recent studies have suggested that in addition to the four major stimuli (iron, inflammation, erythropoiesis and hypoxia) other factors could regulate *HAMP* levels as well [93–101].

#### Growth factors

Growth factors like hepatocyte growth factor (HGF) and epidermal growth factor (EGF) have been shown to inhibit iron and BMP6 mediated induction of HAMP [93]. Treatment of cells with HGF or EGF did not change the pSMAD1/5/8 levels but the amount of pSMAD1/5/8 translocating to the nucleus decreased, hence resulting in reduced downstream signalling [93].

#### Hormones

In addition to growth factors, hormones like oestrogen [94] and testosterone [95–99] have been known to affect *HAMP* synthesis. Treatment of cells with 17β-oestradiol (E2) decreased *HAMP* levels [94], this was shown to be mediated through direct binding to the oestrogen-response elements on the *HAMP* promoter [94]. In another study, it was shown that treatment of HuH7 and HepG2 cells with E2 increases *HAMP* [100]. Unlike the effects of oestrogen, testosterone has been shown to reduce the levels of *HAMP* [96]. Until recently, it was unclear whether this down-regulation is a direct or indirect effect (due to increased erythropoiesis), when it was shown that even in the presence of an EPO neutralizing antibody, testosterone treatment reduced *Hamp* levels in mice [96].

#### Other signalling pathways

The most recent additions to the list of potential pathways regulating *HAMP* have been the Ras–RAF (rapidly accelerated fibrosarcoma) MAPK (mitogen-activated protein kinase) and mammalian target of rapamycin (mTOR) pathways [101]. Using an RNAi screen, components of the Ras–RAF and mTOR pathway were identified as inhibitors of *HAMP* synthesis in HuH7 cells [101]. The Ras–RAF pathway is known to be associated with functions like cell proliferation, cell growth and development, whereas the mTOR pathway is also associated with cell nutrition, oxygen and energy levels [101]. These results emphasize the importance of iron and its regulation, as they link iron metabolism to basic processes like cell growth and cell energetics.

In summary, hepcidin is the key iron regulatory molecule, responsible for the regulation of systemic iron homoeostasis. It is produced predominantly in the liver but can have its effects on cells in distant locations of the body. As illustrated in Figure 1, the regulation of this master iron regulator is complex, with a number of positive and negative regulators. This is probably because of its wide-ranging roles in modulating iron availability for various biological processes and in different disease states. Some of the main regulatory pathways involving iron, inflammation, erythropoiesis, hypoxia, growth factors and hormones have been studied and the mechanisms of regulation deciphered. However, there are likely to be many more additional regulatory factors and pathways that will be uncovered in the future and cement the place of this small molecule as a major player in many homoeostatic processes.

**Figure 1:** Positive and negative regulators of hepcidin BMP6, bone morphogenetic protein 6; BMPR-I, bone morphogenetic protein receptor-I; BMPR-II, bone morphogenetic protein receptor-II; CREB/H, cAMP response-element binding protein/H; EGF, epidermal growth factor; EGFR, epidermal growth factor receptor; EPO, erythropoietin; EPOR, erythropoietin receptor; ERFE, erythroferrone; GDF15, growth differentiation factor 15; HFE, hemochromatosis protein; HIF, hypoxia-inducible factor; HJV, hemojuvelin; IL6, interleukin 6; IL-6R, interleukin 6 receptor; JAK, Janus kinase; PDGF-BB, platelet-derived growth factor-BB; PDGFR, platelet-derived growth factor receptor; SMAD1/5/8, sma and mothers against decapentaplegic homologue 1/5/8 complex; SMAD4, sma and mothers against decapentaplegic homologue 4; STAT3, signal transducer and activator of transcription 3; TFR1, transferrin receptor 1; TFR2, transferrin receptor 2; TWSG1, twisted gastrulation BMP signaling modulator 1.
